The article "GIS-statically-based modelling the groundwater quality assessment coupled with soil and terrain attributes data" was retracted in 2024. Reasons: concerns about the results or conclusions; concerns about the peer review.

# GIS-statically-based modelling the groundwater quality assessment coupled with soil and terrain attributes data

**DOI:** 10.1371/journal.pone.0292680

**Published:** 2023-11-30

**Authors:** Yuwen Chen

**Affiliations:** College of Civil Engineering, Nanjing Tech University, Nanjing, Jiangsu, China; UNITEN: Universiti Tenaga Nasional, MALAYSIA

## Abstract

In this study, we investigated the application of Geographic Information Systems (GIS) for groundwater quality assessment through the integration of statistical models with soil and topographical data. Our primary objectives were to identify soil parameters and topographical attributes contributing to groundwater quality assessment and to evaluate the potential of geostatistics and GIS for spatial analysis of groundwater resources. Groundwater samples were collected from 43 agricultural wells, and surface soil layer samples (0–20 cm) were obtained near each well. We measured groundwater quality parameters and relevant soil properties. Our approach involved the utilization of multiple linear regression (MLR) and principal component regression (PCR), combined with topographical terrain attributes and soil data, for modeling groundwater electrical conductivity (GEC). Our findings revealed significant correlations between GEC and soil electrical conductivity (EC) (r = 0.89) as well as soil carbonate (CaCO_3_) (r = 0.68). Among the ten topographical attributes considered, the terrain wetness index (TWI) exerted the highest influence on GEC (r = 0.57), followed by the slope (r = -0.47). Further analysis demonstrated that the MLR model outperformed the PCR model in both the development and calibration datasets, with an achieved R^2^value of 0.89 and a root mean square error (RMSE)of 150 μScm^-1^ for MLR, compared to an R^2^ of 0.85 and an RMSE of 170 μScm^-1^ for PCR when coupled with soil and attribute data for GEC prediction. The resulting GEC map generated from the MLR model displayed spatial variations, ranging from 605 μScm^-1^ in the northern region to 1275 μScm^-1^ in the central part of the study site. In conclusion, our study demonstrated the effectiveness of combining statistical modeling with geostatistics and GIS for groundwater quality assessment, providing valuable insights for resource management and environmental planning.

## 1. Introduction

Water supply for arid-semi-arid regions like Iran depends heavily on groundwater resources. In addition to that, there are cities and towns without wastewater treatment establishments. Owing to effects such as precipitation, the permeability, and agriculture [1, 2] makes it impossible for wastewater to be utilized and recycled for other purposes [3]. Several provinces in Iran’s south, which have semi-arid and arid climates, rely on groundwater as their primary source of fresh water for irrigation [4, 5]. In recent decades due to population growth, the amount of groundwater used by humans has increased in a considerable manner. This includes drinking, agriculture, industry, and many other purposes, making wastewater treatment challenging. These impacts on the downstream environment and groundwater are complicated [6]. To better manage groundwater reservoirs, it is imperative to analyze groundwater quality in addition to monitoring the groundwater levels [3–7]. To accurately measure groundwater quality for various components related to groundwater, conventional methods are commonly used to obtain an indication of a particular parameter as well as its complexity. Generally, these methods involve a considerable amount of time, money, and labor and require a lot of expertise. Some regions also present difficulties in sampling groundwater. The lithology, morphology, soil formation related to groundwater health, slope, dam construction and topography of the land are generally associated with groundwater quality [8–10]. Therefore, new big-data analyses are required to analyze groundwater, since traditionally, environmental data is interpreted using statistical models [3, 7, 11].

The article "GIS-statically-based modelling the groundwater quality assessment coupled with soil and terrain attributes data" was retracted in 2024. Reasons: concerns about the results or conclusions; concerns about the peer review.

Because the pH of groundwater is relatively constant in Iran aquifers because carbonate formations are abundant in the majority of the country, particularly in the southern lands, it cannot function as a reliable indicator of groundwater quality [5, 12]. However, some research groups have tried to use this indicator as a measurement of potential groundwater quality. For example, Osman et al. [13] found declining groundwater levels in Malaysia. They developed a predictive statistical model based on 11 months of data. This model outperformed others, especially when considering 1-day delayed groundwater levels as input (R^2^ = 0.92). Their study sets a strong benchmark for groundwater quality predictions in the future. Irwan et al. [14] emphasized the critical role of water in agriculture and daily life, highlighting its impact on various aspects. They reviewed 83 studies from 2009 to 2023, focusing on water quality prediction methods and artificial intelligence models. They discussed the potential of generative adversarial networks (GANs) and transformers to improve water quality prediction by addressing data limitations. In areas with a wide range of electrical conductivity (EC), groundwater EC is a better index of groundwater quality. The development of statistical models is possible since simple assessments of groundwater quality cannot suffice for various purposes, particularly at large scales where lots of sampling wells are present. Besides the common linear regression method, principal component (PC) regression is also a reliable approach for examining groundwater quality [6–8]. The MLR method is used to develop forecasting models based on the results of the PCR to find relationships between quality parameters. Moreover, MLR is useful for determining whether one or more variables are more important, as well as for identifying outliers and anomalies. Because GIS provides readily suitable methods for manipulating spatial data, groundwater quality can now be evaluated quickly and efficiently using GIS as a visual tool [3, 4]. Statistical modeling and groundwater quality are integrated to successfully map, manage and protect groundwater.

The article "GIS-statically-based modelling the groundwater quality assessment coupled with soil and terrain attributes data" was retracted in 2024. Reasons: concerns about the results or conclusions; concerns about the peer review.

Combining statistical modeling, geostatistics, and GIS for groundwater quality assessment offers numerous advantages [1, 15]. It enables the visualization of spatial trends, the integration of diverse data types, and the generation of accurate groundwater quality maps. This integrated approach also supports data validation, decision-making, and risk assessment. Furthermore, it facilitates the comprehension of temporal fluctuations and trends in groundwater quality. This approach has a wide range of potential, including environmental management, water resource planning, contamination detection, public health evaluation, and more. It aids in informed decision-making and resource management across various sectors. However, accurate results of this combination rely on data quality and availability, demanding high-resolution data and expertise. Model complexity affects predictability, and validation can be challenging with limited data. It may not fully address short-term changes or causality but remains a valuable tool for groundwater quality management when used judiciously.

The GIS and statistical methods have been combined in several studies to analyze spatial groundwater quality [16–18]. A GIS technic integrated with a statistical approach was documented by Haghizadeh et al. [3] for analyzing the groundwater in the Broujerd region of Iran. Eleven quality factors were obtained from DEM for mapping groundwater. A study conducted by Yadav et al. [19] highlighted a combination GIS with PCA to identify the contaminants of aquifers in India. Their findings pointed out that PCA coupled with a GIS tool provides acceptable results for the assessment of groundwater. According to Naghibi et al. [20], a groundwater quality map of Koohrang, Iran was generated using data mining, considering 13 environmental factors. They found that the integration of environmental data with data-mining approaches could provide valuable insight into the potential quality of groundwater. GIS-AHP was used by Shahid et al. [18] for assessing groundwater quality in the Western Ghats, India. The results of their study indicated that the method was approximately 85% accurate. As part of an investigation into groundwater quality in rural northwest Iran, Mosaferi et al. [21] employed PCA together with a GIS. They reported that multivariate analysis could be successfully applied to the evaluation of groundwater. Honarbakhsh et al. [11] found that the combined use of geostatistics and geographic information systems (GIS) provided acceptable results for assessing groundwater quality. Abdalla et al. [22] demonstrated that the integration of RS and GIS leads to improving the monitoring of water resources. In Pakistan, Ijumulana et al. [23] highlighted the potential risks of groundwater in GIS. They indicated that drinking water quality varied from one geological to another.

The article "GIS-statically-based modelling the groundwater quality assessment coupled with soil and terrain attributes data" was retracted in 2024. Reasons: concerns about the results or conclusions; concerns about the peer review.

Despite the benefits of the use of GIS to investigate groundwater quality, few researchers have merged GIS and statistical models to evaluate groundwater in southern Iran. Statistical analysis coupled with GIS has not been utilized for assessing the relationships between soil, topographical attributes, and groundwater. Also, the effects of geological terrain attributes on the quality of groundwater have not been adequately examined. The aims of this therefor research were: (1) to test the statistical attitudes (PCR and MLR) for evaluating the groundwater quality in Firuzabad, Iran, which is a main water source for drinking and irrigating purposes water. In addition, we attempted: (1) to identify soil parameters and topography attributes that can be used to assess groundwater quality, and (2) to evaluate the potential of a GIS application to analyze the spatial analysis of groundwater potentials.

## 2. Materials and methods

### 2.1. Study site and sampling

The study area is situated at a latitude and longitude of 28°52′ to 28°47′ N and 52°24′ to 52°39′ E in Firuzabad, Fars, Iran (Fig 1). The aquifer acreage is 282.5 km^2^ (Fig 1) of Firuzabad plain with an area of 545 km^2^. Firuzabad Aquifer is the main source of drinking water for the city of Firuzabad with 121,000 and approximately 25 villages. Furthermore, it provides irrigation water for agricultural purposes. The climate at the region is semi-arid with 291.7 mm of rainfall and 17.5°C. The wettest months are December, January, and February. Summer months are marked by high temperatures, while winter months are marked by relatively low temperatures. An altitude range of 1124–2721 m was observed. At the center of the area, there are agricultural lands, whereas the elevated areas are dominated by mountains. Alluvial deposits dated between Q1 and Q3 are dominated by dolomite and calcite [4, 11]. The marls and limestones in both the Hormuz and the Asmari are also soluble [11]. The Inceptionsol, the Entisol, and the Aridisol (Soil Taxonomy) are three types of soil. The water was found 45 meters below ground level [24].

The article "GIS-statically-based modelling the groundwater quality assessment coupled with soil and terrain attributes data" was retracted in 2024. Reasons: concerns about the results or conclusions; concerns about the peer review.

**Fig 1:** Study site. Original maps generated in GIS.

### 2.2. Soil and groundwater sampling

Groundwater samples were collected from 43 agricultural wells. The location of the wells was recorded using a portable GPS. EC was modeled for 43 agricultural wells in Firuzabad to assess the potential quality of groundwater. The study did not involve private land, protected land, endangered or protected species. No specific permissions were required for these locations/activities. We measured the electrical conductivity of the samples using a portable EC meter. In addition to groundwater samples, we also collected 1 kg of topsoil (0–20 cm) near the studied wells. The hydrometer method was utilized for the dried, and sieved samples for lab measurements [25], calcium carbonate was neutralized with 1 normal HCl, and EC and pH of soil samples were measured using EC/pH meters at different depths using EC meters. Soil texture was obtained using the hydrometer. Soil organic matter (SOM) was determined using the Walkley-Black method [26].

### 2.3 Methodology

Fig 2 depicts the methodology approach of this study. Maps of soil properties were generated using Ordinary Kriging (OK). There is widespread use of this method to assess groundwater quality [27], and the variogram in ArcGIS 10.6 shows good performance [28].

$$\beta \left(\text{T}\right)=\frac{1}{2\text{N}\left(\text{T}\right)}\sum_{\text{i}=1}^{\text{N}\left(\text{h}\right)}{\left[\text{K}\left({\text{x}}_{\text{i}}\right)-\text{K}\left({\text{x}}_{\text{i}}+\text{T}\right)\right]}^{2}$$ (1)

$$\hat{\text{K}}\left({\text{x}}_{\text{i}}\right)=\overset{\text{N}}{\underset{\text{i}=1}{\sum }}\;\lambda_{\text{i}}\text{K}\left({\text{x}}_{\text{i}}\right)$$ (2)

where K(x_i_), β(T), and N(T) are independent components, the variogram from K(x_i_) to K(x_i_ + T). Various attributes have been introduced as input layers for modeling groundwater quality in GIS, including slope (Fig 3a), aspect (Fig 3a), profile curvature (P_Cur), flow direction (FD), plan curvature (Pl_Cur), flow accumulation (FA), LS factor (Fig 3c), and topographic wetness index (TWI) (Fig 3d). To determine soil erosion, sedimentation, and redistribution (Table 1) [20], length-slope factors, stream power factors, and sediment transport factors have been used (Table 1) (Liu et al.). The topographic parameters were generated from a Digital Elevation Model (DEM) provided by the USGS. ArcMap v.10.6.2 was used to create maps of elevation and study site. The slope and aspect modules in the SAGA 2.2.5 were used to calculate curve metrics (P_Cur and Pl_Cur). Stream power index and length-slope factor were generated in SAGA using the SPI and LS-factor modules. The SAGA TWI was used to calculate catchment area (m^2^) and TWI. The filtered DEM was used to extract flow direction and flow accumulation maps. All the topography attributes are illustrated in Table 1.

The article "GIS-statically-based modelling the groundwater quality assessment coupled with soil and terrain attributes data" was retracted in 2024. Reasons: concerns about the results or conclusions; concerns about the peer review.

**Fig 2:** Flow chart of the methodology.

**Fig 3:** Aspect (a), slope (b), LS factor (c), and topography wetness index (d) of the studied site.

**Table 1:** Definitions, formulas and significances of selected topographic factors.

Variables	Definition	Formula	Significance	References
Elevation (h)	Height from see level	―		
Slope (S) (radian)	An angle between a tangent and a horizontal planes at a given point	$S=arctan\sqrt{p^{2}+q^{2}}$	Velocity of runoff and soil-water content	Li et al. [29]
Aspect (A) (radian)	An angle clockwise from north to the horizontal projection of an external normal vector at a given point	$A=arctan\left(\frac{q}{p}\right)$	Soil-water balance, vegetation distribution	Li et al. [29]
Profile curvature (m ^-1^)	Curvature of the surface in the direction of the steepest slope	$k_{v}=-\frac{p^{2}r+2pqs+p^{2}t}{\left(p^{2}+q^{2}\right)\sqrt{1+p^{2}+q^{2}}}$	Flow convergence and divergence, soil- water content	Tucker and Bras [30]
Plan curvature	Curvature in a horizontal plane	$k_{h}=-\frac{q^{2}r+2pqs+q^{2}t}{\left(p^{2}+q^{2}\right)\sqrt{1+p^{2}+q^{2}}}$	Flow convergence and divergence, soil water content	Tucker and Bras [30]
Catchment area (m^2^)	Area draining to the catchment outlet	―	Runoff velocity and volume	Moore et al. [31]
Flow accumulation (FA)	Upslope number of grid cells	―	Soil-water content and runoff volume	Mirzaee et al. [28]
Topographic wetness index (TWI)	Frequencies and duration of saturated conditions	$TWI=\text{ln}\left(\frac{A_{S}}{S}\right)$	Soil moisture distribution	Wilson and Gallant [32]
Length-Slope factor (LS)	Erosive power of the terrain	$LS=\left(n+1\right)STI=\;{\left(\frac{A_{S}}{22.13}\right)}^{0.4}{\left(\frac{\text{sin}\;\theta }{0.0}\right)}^{1.3}$		Moore et al. [31]
Stream power index (SPI)	Erosive power of overland flow	*SPI* = *A*_*s*_ tan *θ*	Soil erosion, convergence of flow	Wilson and Gallant [32]; Mirzaee et al. [28]
Sediment transport index (STI)	Soil-water content and sediment transport	$STI=\;{\left(\frac{A_{S}}{22.13}\right)}^{0.4}{\left(\frac{\text{sin}\;S}{0.0896}\right)}^{1.3}$	Soil erosion and deposition	Wilson and Gallant [32]; Mirzaee et al. [27]

Where p, q, r, and t are partial derivatives of elevation (h): $h=f\left(x,y\right);p=\frac{\delta h}{\delta x};q=\frac{\delta h}{\delta y};r=\frac{\delta^{2}h}{\delta x^{2}};t=\frac{\delta^{2}h}{\delta y^{2}}$

Fig 4 illustrates maps of groundwater EC (GEC) (a), groundwater HCO_3_ (b), groundwater total hardness (TH) (c), groundwater chloride (Cl) (d), soil EC (e), and soil CaCO_3_. As can be seen in Fig 4a–4d, groundwater EC, HCO_3_, and Cl had the same trend, with the highest amount of the parameters found in the central area where the geological formation is limestone. Interestingly, the map of the soil EC is similar to the GEC. A variation in soil CaCO_3_ can be seen in Fig 5a from 21% in the north to 47% in the south of the site. The spatial variation of SEC and GEC in the study site was very similar (Fig 4a and 4f). An area with soluble materials showed the highest EC values in soil and groundwater. Fig 4a and 4f indicate that GEC and SEC are widely distributed in this study site. CaCO_3_ and EC in groundwater increased at the study site as a result of soluble carbonate formation.

The article "GIS-statically-based modelling the groundwater quality assessment coupled with soil and terrain attributes data" was retracted in 2024. Reasons: concerns about the results or conclusions; concerns about the peer review.

**Fig 4:** Spatial map of groundwater EC (a), groundwater HCO_3_ (b), groundwater TH (c), groundwater Cl (d), soil EC (e), and soil CaCO_3_ (f).

**Fig 5:** Semi-variograms for soil and groundwater EC.

In order to address the non-uniform units issue, all topographic variables were standardized before modeling. Furthermore, the data were tested for normality before modeling. There were 43 wells in total, 30 wells were selected for model development by random selection and 13 wells were selected for model validation. We conducted a *t*-test (p<0.05) to determine whether there were significant differences between the two data sets. The GEC and topographic variables, as well as soil properties, were investigated for the correlation using Pearson test analyses (p< 0.05). As a result, of the selection of significant topographical variables, a stepwise MLR (SMLR) was employed for the prediction of GEC as follows:

$$\text{GEC}=\text{B}+{\text{b}}_{1}{\text{X}}_{1}+{\text{b}}_{2}{\text{X}}_{2}+{\text{b}}_{3}{\text{X}}_{3}+\ldots +{\text{b}}_{\text{N}}{\text{X}}_{\text{N}}.$$ (3)

b_1_ to b_N_ represent regression coefficients, X_1_ to X_N_ represent input variables, and X_1_ to X_N_ are GEC. In order to test multicollinearity [24], the VI (Variance Inflation) Factor was utilized [33]:

$$\text{VIF}=\frac{1}{1-{\text{R}}_{\text{j}}^{2}}$$ (4)

If VIF is greater than 5, this indicates collinearity between input variables [24]. Statistica 8.0 was used to complete the MLR. PCR (principal component regression) was performed using Statistica 8.0 software in order to eliminate collinearity, diminish the dimension of data sets, and reduce input variables. At least 85% of the variance in the original data set could be explained by the principal components (PCs) [25]. We then set up PCs as independent variables for the modeling. Eq (5) is used for rescaling the input variables and the EC. Rescaled data is Xn, and observed data is Xmin and Xmax. To evaluate MLR and PCR, RMSE (root mean square error) R^2^, and ME (mean error) were used as follows:

$${\text{R}}^{2}=\frac{{\left[\sum_{\text{i}=1}^{\text{n}}\left({\text{O}}_{\text{i}}-\bar{{\text{O}}_{\text{i}}}\right)\;\left({\text{P}}_{\text{i}}-\bar{{\text{P}}_{\text{i}}}\right)\right]}^{2}}{\sum_{\text{i}=1}^{\text{n}}{\left({\text{O}}_{\text{i}}-\bar{{\text{O}}_{\text{i}}}\right)}^{2}\;\sum_{\text{i}=1}^{\text{n}}{\left({\text{P}}_{\text{i}}-\bar{{\text{P}}_{\text{i}}}\right)}^{2}},$$ (5)

$$\text{RMSE}=\sqrt{\left(\frac{\sum_{\text{i}=1}^{\text{n}}{\left({\text{P}}_{\text{i}}-{\text{O}}_{\text{i}}\right)}^{2}}{\text{n}}\right)},$$ (6)

$$\text{ME}=\frac{\sum_{\text{i}=1}^{\text{n}}\left({\text{P}}_{\text{i}}-{\text{O}}_{\text{i}}\right)}{\text{n}}$$ (7)

where n represents the measurements, O represents the measured parameters, P represents the predicted parameters, and i is the parameter [19].

The article "GIS-statically-based modelling the groundwater quality assessment coupled with soil and terrain attributes data" was retracted in 2024. Reasons: concerns about the results or conclusions; concerns about the peer review.

## 3. Results and discussion

### 3.1 Soil properties

The soil properties are summarized in Table 2. A Kolmogorov-Smirnov test, however, found that properties were normally distributed. According to the USDA classification system, the majority of samples were classified as loams, silty clay and, loams clay loams. It is estimated that 41.22 percent of soil particle size is attributed to silt content. There was a mean calcium carbonate content of 44.4%, which ranged from 11.60% to 57.70%. A minimum value for OM is 0.94%, a maximum value is 4.49%, and a mean value of 1.82%. Ostovari et al. [33] found that organic matter levels were similar to those in Semikan, which has a similar climate. EC values of soils varied from 1350 to 1983 μS cm^-1^ and pH values range from 7.14 to 8.15. The soil is likely to be calcareous since most Iranian soils have high CaCO_3_ contents.

**Table 2:** Mean, minimum, maximum of soil samples.

Parameter	Mean	Min	Max	Std	cv
pH	7.78	7.14	8.18	0.23	4.25
EC (μS cm^-1^)	1350	854	1983	72.88	19.69
BD (g cm^-3^)	1.43	1.24	1.83	0.26	10.20
%Sand	30.45	1.02	86.26	12.48	16.33
%Clay	27.32	5.24	56.43	10.70	21.73
%Silt	41.22	8.61	75.73	13.74	36.25
%CaCO_3_	38.40	11.60	47.70	11.59	26.10
%SOM	1.82	0.94	4.49	0.64	32.38

Videography analysis of soil EC, CaCO_3_, GEC and groundwater HCO_3_ are presented in Table 3 and Fig 5. All variograms are anisotropies. In terms of soil and groundwater properties, the spherical models performed best (Table 2). There is a positive link exists between GEC and soil CaCO_3_, indicating that carbonate elements (Ca^2+^ and Mg^+2^) have a notable influence on GEC. Table 2 shows that C0/sill is strong to moderate dependent (0.10–0.67) [27]. There was a good agreement between soil maps and OK [28]. It appears that groundwater EC is strongly spatially dependent, as indicated by a spatial dependency of 0.10 for the spherical model. As presented in Table 3, the ordinary kriging (OK) method with R^2^ between 0.65 and 0.76 showed a good performance in the spatial prediction of soil and groundwater quality (Table 3). The soil EC was found to be significantly affected by CaCO_3_, indirectly affecting the groundwater EC reported by Ostovari et al. [33]. Increasing the salinity of groundwater may be caused by the formation of carbonate due to the high concentration of soluble materials [34]. The water type in the Firuzabad groundwater is Na-Cl based on TDS values of 1800 mgL^-1^ and EC values of 1983 μS cm^-1^. Ca^2+^ and Mg^2+^ have a vital role because of the presence of carbonate formations with a large quantity of dolomite, as reported by Honarbakhsh et al. [4]. Firuzabad River drains lots of urban sewage with high chloride that can reduce the water quality. As a result of weathering, carbonite formations dissolve in semiarid aquifers.

The article "GIS-statically-based modelling the groundwater quality assessment coupled with soil and terrain attributes data" was retracted in 2024. Reasons: concerns about the results or conclusions; concerns about the peer review.

**Table 3:** Semi-variograms information and kriging method.

Parameters	Model	Nugget/Sill	Range (m)	Sill	Nugget	R^2^	RMSE	ME
GEC	Spherical	0.10	6800	27100	2650	0.65	0.991	0.153
HCO3	Spherical	0.14	6350	415	56	0.68	3.224	−0.034
Soil EC	Spherical	0.12	8100	23300	2700	0.76	2.115	0.024
Soil CaCO3	Spherical	0.67	3920	17	58	0.75	2.228	0.064

### 3.2. Development of MLR model

The correlation between topography attributes and GEC and soil-EC was investigated using Pearson test as given in Fig 6. %CaCO_3_ had a significant correlation with both GEC and soil EC, indicating the impact of the carbonate formation on both soil and groundwater quality. In general, terrain attributes are more correlated with soil EC than with GEC. Many topographic attributes were strongly interrelated, making them impossible to consider independent variables. We found a significant association between TWI, aspect, FA, and STI. The main variables affecting GEC were identified through PCA. According to Table 4, 73% of the variability in topographic attributes can be attributed to the first four PCA components. The most significant terrain attributes for PC1 were TWI, Slope, P_CU, FL, and LS-factor. PC2 is influenced by elevation, SPI, and FA factors. Elevation may not influence soil erosion and deposition, despite having a loading score of -0.619 (Fig 6). Possibly due to the similar altitude at which the samples were collected. Several attributes (including STI, TWI, and aspect) were significantly positively correlated with GEC. Significantly negative correlations were found between slope GEC, while significant positive correlations were found between TWI and FD. Li et al. [29] found that TWI was positively correlated with soil properties. TWI is useful for studying soil-water content variations along slopes [29]. TWI determines soil moisture gradients. There was a positive correlation between TWI and GEC and soil EC, indicating that saturated soil tends to accumulate these compounds. The TWI values were higher in landscapes with lower elevations.

The article "GIS-statically-based modelling the groundwater quality assessment coupled with soil and terrain attributes data" was retracted in 2024. Reasons: concerns about the results or conclusions; concerns about the peer review.

**Fig 6:** Correlation matrix of GEC and soil and topographical attributes.

**Table 4:** Loading score of the PCs for topographic attributes.

	PC1 (33.4%)	PC2 (15.6%)	PC3 (14.2%)	PC4 (9.8%)
Aspect	-0.222	0.069	0.535	0.478
Flow_accu	0.486	-0.600	-0.142	0.076
Elevation	-0.356	-0.619	0.395	-0.020
Watershed	-0.132	-0.001	-0.059	-0.377
Slope	-0.687	-0.266	-0.262	0.021
Pl_cu	-0.525	0.265	-0.243	0.415
Flow_lengh	-0.521	-0.511	-0.130	-0.140
P_cu	0.475	-0.099	0.043	-0.642
Basin	-0.087	-0.345	0.735	-0.162
STI/LS	0.457	-0.525	-0.277	0.385
SPI	-0.227	0.624	0.226	-0.175
TWI	0.698	0.053	0.411	0.294

Table 5 presents the results of the MLR model based on soil-topographical parameters. According to MLR, groundwater EC was significantly correlated with Soil EC, slope, CaCO_3_, flow length and TWI. As given in Table 5, the most controlling parameters in the GEC prediction were soil EC with Beta of 0.78, followed by %CaCO_3_ with Beta of 0.65, and TWI with Beta of 0.53. Due to soil calcareousness, CaCO3 is an important factor for groundwater quality. Slope and the flow length both showed significant effects at p 0.05. TWI and CaCO_3_ showed significant positive effects at p 0.001. Based on the linear model, the following equation can be obtained:

GEC=23654+0.48SoilEC–17.22Slope+87.25CaCO3+145..66TWI+2541Flowlength (8)

where GEC and SEC (μS cm^−1^), respectively, CaCO_3_ represents soil carbonate (%) and TWI illustrates the topography wetness index. LS factor and TWI played a significant role for the groundwater quality modeling according to Haghizade et al. [3] and Naghibi et al. [20]. Table 5 indicates no multicollinearity among input variables. A number of topographical factors, particularly TWI, have been shown to have an impact on the hydrological process of soils and water [28].

**Table 5:** The MLR details for the prediction of GEC.

Parameter	Beta (Standardized Coefficients)	Std. Err.	Unstandardized Coefficients B	Significance	VIF
Intercept			23654.32	0.020	3.2
Soil EC	0.78	0.04	0.48	0.000	3.5
CaCO_3_	0.65	0.04	87.25	0.000	2.8
Slope	−0.21	0.04	−17.22	0.034	2.6
Flow length	0.15	0.03	2541.35	0.021	4.5
TWI	0.53	0.03	145.66	0.001	3.6

The article "GIS-statically-based modelling the groundwater quality assessment coupled with soil and terrain attributes data" was retracted in 2024. Reasons: concerns about the results or conclusions; concerns about the peer review.

### 3.3. PCs analysis

PC1 with r = 0.698 was positevely correlated with GEC, followed by PC2 with r = 0.42. Aspect, SPI, and STI factors contributed 15.6% of variance (Table 4). Fig 7b shows the influential factors influencing the GEC, including SPI, slope, LS factor, and elevation. The TWI with loading score 0.411 and aspect with loading score 0.535 defined PC3 with an 9.8% variance. Based on the four first PCs, the following regression model predicts groundwater EC:

$$\text{GEC}=4230.5+2563.6\;\text{PC}1+290.5\;\text{PC}3+1264.7\;\text{PC}2\;{\text{R}}^{2}=0.78$$ (9)

**Fig 7:** Loading score of PC1–PC2 (a) and PC1–PC3 (b).

Groundwater EC is represented by GEC. Using Eq (9), PC1 with Beta = 0.74 and PC2 with Beta = 0.41 were considered as significant variables. Even though PC4 was considered one of the input variables, the model did not include it. Fig 8 depicts that both the MLR and PCR are fitting nicely on the basis of the residual plot. Positive residuals (y-axis) indicate that the estimation was significatly low; negative residuals indicate that it was too high; zero indicates that it was exactly correct. Fig 8 shows most points are around the X line, indicating the estimation was correct. Estimated GEC in both development and validation data sets versus the observed GEC is given in Fig 9. Fig 9a and b detemin how the PCR significatly underestimated the GEC. Contrary to what was observed for the PCR model, the MLR predicted GEC with better performance (Fig 9a, 9b). On the basis of soil topographic parameters as a prediction tool, MLR performed better than PCR for the estimation of GEC. The statistical criteria for the MLR model (R^2^ = 89, RMSE = 150 and ME = 45) were better than those for PCR model (R^2^ = 85, RMSE = 170 and ME = 51) in both development and validation data-sets. MLR can predict groundwater EC with an accuracy of 95%, according to Saleem et al. [35] and Kamakshaiah and Seshadri [36]. Yadav et al. [19] documented the performce of the GIS integrated with PCA to investigate the quality of groundwater in India. Several researchers have shown that PCA models are more accurate at predicting groundwater quality, including Elizabeth et al. [37]. According to Van-Westen et al. [38], it is critical that bivariate statistical models do not assume conditional independence. The models are particularly useful for determining groundwater potential in specific locations. Moreover, Pradhan et al. [39] highlighted animportant disadvantage of statistical models: it is difficult to distinguish between significant factors. Each finding, therefore, may experience different drawbacks based on different circumstances.

The article "GIS-statically-based modelling the groundwater quality assessment coupled with soil and terrain attributes data" was retracted in 2024. Reasons: concerns about the results or conclusions; concerns about the peer review.

**Fig 8:** Residual prediction of both (MLR and PCR) estimation models.

**Fig 9:** Measured GEC VS predicted GEC for both (MLR and PCR) estimation models in calibration (a) and validation (b) sets.

The GEC spatial variability (Fig 10) was depicted using GIS on the basis of the formulated MLR model. The GEC values varied from 605 in the north-east to 1275 μScm^−1^ in the center of the area (Fig 10). According to the Fig 10, only 21% of the Firuzabad Aquifer had EC more than 1000 μScm^−1^, which is moderately appropriate for the agricultural crops in Firuzabad Plain. While, the rest of the area (79%) had EC < 1000 μScm^−1^, indicating a suitable groundwater crop production (Fig 10). A GIS joined with statistical models has been reported for the evaluation of groundwater quality in Iran [3+6]. Consequently, soluble chalky-carbonate formation in the center of Firuzabad affects groundwater, resulting in higher soluble salt levels (total dissolved solids). Based on the MLR developed model, the spatial variability of groundwater ECs (Fig 10) is very similar to that of the soil ECs (Fig 4f). Honarbakhsh et al. [4] also pointed out that a region with the highest groundwater quality risk was located in the center of Marvdasht Plain, where groundwater flow convergence occurs. Based on the Kappa index of 0.75, the MLR model and the Kriging method provide a good match for the GEC map. It is worth mentioning that statistical methods for assessing the quality of groundwater have some uncertainties. A situation of uncertainty refers to uncertainty regarding the outcome of an event. There may be a number of explanations for the lack of confidence, such as incompleteness, blurriness, accuracy, unreliability, inconclusiveness, or potential falsity in the information.

**Fig 10:** Spatial variability of the GEC generated from the MLR model.

## 4. Conclusions

GIS-based groundwater quality assessments can be valuable for providing valuable insight into these resources’ potential quality using statistical models and soil and topographical data. To evaluate groundwater quality, we examined soil parameters and topographic attributes. Moreover, we examined how geostatistics and geographic information systems could be used to analyze groundwater potential spatially. There was a significant correlation between soil EC and soil carbonate (CaCO3) with GEC of 0.89 and 0.68, respectively. The typography wetness index (TWI) had a correlation coefficient of 0.57, while the slope had a correlation coefficient of -0.47 among the 10 topographical attributes. MLR had better performance (R^2^ = 0.89 and RMSE = 150 μScm^-1^) coupled with soil and attributes data in both development and calibration data sets than PCR (R^2^ = 0.85 and RMSE = 170 μScm^-1^). GEC in the study site ranged from 605 μScm^-1^ in the north to 1275 μScm^-1^ in the center, according to the GEC map generated by the MLR model. Based on our research, we concluded that statistical modeling combined with geostatistics and geographic information systems can produce satisfactory results for the assessment of groundwater quality. We also recommend improving the effectiveness of this approach by expanding data collection efforts to include high-resolution spatial data to enhance model accuracy. Additionally, integrating advanced machine learning techniques alongside traditional statistical methods and geostatistics can capture complex relationships and enhance predictive power.

The article "GIS-statically-based modelling the groundwater quality assessment coupled with soil and terrain attributes data" was retracted in 2024. Reasons: concerns about the results or conclusions; concerns about the peer review.

## Supporting information

S1 Data (XLSX)
